# Computed Tomography Image Segmentation Algorithm to Detect the Curative Effect of Radial Shock Wave Therapy for Knee Osteoarthritis

**DOI:** 10.1155/2021/7098924

**Published:** 2021-08-05

**Authors:** Jinghai Tian, Guoyong Chen, Fuhong Peng, Guotang Lan

**Affiliations:** ^1^Department of Orthopedics, People's Hospital of Dongxihu District, Wuhan 430030, Hubei, China; ^2^Department of Orthopedics, Wuhan Asia Heart General Hospital, Wuhan 430000, Hubei, China; ^3^Department of Orthopedics, Tongji Hospital, Tongji Medical College, Huazhong University of Science and Technology, Wuhan 430000, Hubei, China

## Abstract

The aim of this study was to investigate the values of computed tomography (CT) imaging technology based on image segmentation algorithm (ISA). It was applied in the radial shock wave therapy (RSWT) to treat knee osteoarthritis (KOA), so its curative effect and rehabilitation effect on nerve function were mainly analyzed in this study. 84 patients with KOA were selected and grouped into an ultrasonic treatment group (group A) and a RSW group (group B). All the patients received the ISA-based CT examination and high-quality nursing intervention. There were comparisons on the effects of pain improvement, knee joint function, and nerve function rehabilitation of patients in groups A and B. Results showed that visual analogue scale (VAS) scores before and after treatment were markedly different among all patients, and the pain degree of patients in group B was lower than the degree of group A (*P* < 0.05). The knee joint function of group B after treatment was greatly better than group A (*P* < 0.05). Scandinavian stroke scale (SSS) scores of nerve function rehabilitation after nursing in patients from group B were sharply lower than the scores of group A (*P* < 0.05). Results indicated that ISA-based CT images could be applied in analysis of curative effect on KOA, and there was more obvious effect of RSWT in the treatment of KOA.

## 1. Introduction

KOA is a relatively common type of chronic osteoarthritis, which accounts for about 6% of all osteoarthritis [1]. The incidence of KOA is related to age; namely, the higher the age, the higher the incidence of KOA [2]. Studies have shown that the incidence of KOA in people who have been in semisquat or kneeling positions for a long time, such as underground coal miners and construction workers, is higher than that in the normal population [3]. KOA is usually caused by degeneration of the knee joint, overwork, trauma, and other factors, but the specific pathogenesis is not clear. Besides, RSWT is a common treatment for bone diseases [4]. It is mainly employed to collect a variety of acoustic energy single fluctuations into the focus area of targeted tissues by inducing energy convergence and to achieve a variety of therapeutic stimuli of different degrees by applying angle and pressure adjustment. RSWT is very effective in relieving pain and treating bone diseases such as supracondylar, calcified tendonitis, and plantar fasciitis [5, 6]. In addition, RSWT is a noninvasive treatment with minimal trauma and relatively few complications for patients, which does not require hospitalization. As a result, the economic pressure on patients is greatly reduced, so it is widely applied in clinical treatment. Therefore, as a treatment method with little trauma and side effects, RSWT has a very critical clinical significance in the treatment of KOA.

CT imaging is an effective method for the clinical diagnosis of KOA [7]. CT imaging can clearly observe the osteoarthritis lesions of knee joint, thus providing a strong help for the diagnosis and follow-up treatment of doctors [8]. In recent years, the resolution of medical image is constantly improved with the rapid development of modern medical image technology, while the traditional segmentation technology is difficult to obtain satisfactory segmentation results. Image segmentation is a critical step for image analysis and three-dimensional reconstruction in medical imaging, and the realization of accurate segmentation helps doctors understand the actual condition of patients and make reasonable treatment plans [9, 10]. Image segmentation technology based on graph theory is a hot research topic in the image segmentation in recent years [11]. It not only emphasizes global constraints, but also pays special attention to local information processing, so the segmentation results are better than those of traditional segmentation methods. The regions or pixels in the original image based on ISA are interpreted as nodes in the graph, transforming medical image segmentation into the graph-based energy minimization and dealing with the application of maximum flow/minimum segmentation algorithm [12]. Thus, ISA was used for image segmentation processing of CT imaging techniques and applied in the analysis of curative effect of RSWT for KOA. Through the analysis of pain symptoms before and after treatment, the knee joint function, and nerve function recovery, there was a theoretical basis for the clinical diagnosis and treatment of KOA.

## 2. Materials and Methods

### 2.1. Subjects Investigated and Grouping

84 patients with KOA were selected as the subjects investigated, who were admitted to hospital from October 2018 to May 2020, including 46 males and 38 females. All patients were rolled into the ultrasound treatment group (group A) and RSW group (group B) based on different treatment methods, with 42 cases in each group. The ethics committee of the hospital had approved this experiment, and all the subjects included in this experiment had known and agreed.

The criteria for inclusion were defined to include patients who were diagnosed with KOA, were older than 42 years and younger than 70 years, had been informed and agreed, and had complete clinical data.

The criteria for exclusion were defined to include patients who suffered from severe heart, brain, and hematopoietic diseases, mental illness, knee joint infection, tumor, or rheumatic immune system diseases, were in the pregnant and lactating period, and had contraindications for ultrasound or RSWT.

### 2.2. Therapeutic Methods

The patients of group A were given ultrasonic treatment. Coupling agent was applied to the head of the ultrasonic arthritis treatment instrument, so as to treat the pain points around the knee joints. The intensity was set at 1.0–1.2 W/cm during the treatment, and the ultrasonic arthritis treatment instrument was first moved around pain points at a constant speed of 5 minutes with a speed of 5 mm/s. Then, the fixed treatment was for the pain points of the knee joints for 10 minutes. The treatment was once a day, five times a week for a four-week course.

The patients of group B were treated with RSWT apparatus. The impact points of knee pain points and calcification were selected according to the imaging data of patients. 7 treatment points were selected for each treatment, and each point was impacted 600−800 times. The output pressure was set as 2.5–3.5 bar, and the frequency was within the range of 10−15 Hz. The interval of each treatment was 5 days, and 5 consecutive treatments were regarded as a course of treatment. Besides, adverse reactions were observed and recorded during the treatment.

### 2.3. Computed Tomography Examination

All patients were examined by CT imaging and the instrument was Philips 128-slice spiral CT. The specific examination method was as follows. The patient was placed in the supine position and the flat foot was first entered. Then, the local position of the knee joint was scanned, the layer thickness was set at 0.6 mm, the layer spacing was set at 2 mm, and the pitch parameter was 1.0. The data were uploaded to the workstation for coronal and sagittal reconstruction after the scanning.

### 2.4. Computed Tomography Imaging Technology Based on Image Segmentation Algorithm

Graph Cuts algorithm fused all the information of the global and local images and fully reflected the correlation of image pixels, so it has marked advantages in the image segmentation. Graph Cuts algorithm input source image and corresponding label. Suppose that there was *l* ∈ {0,1} marked by any pixel point *q* of the image, and 0 represented the background and 1 stood for the foreground. In order to obtain the best binary segmentation result, the expression of the quantity function was defined as follows:

(1) $$\begin{array}{c} E\left(L\right)=\lambda *\sum_{p\in N}R_{p}\left(l_{p}\right)+\sum_{\left\{p,q\right\}\in N}A_{\left\{p,q\right\}}\cdot \delta \left(l_{p},l_{q}\right). \end{array}$$

There were two equations below to supplement and explain (1):

(2) $$\begin{array}{c} \left\{\begin{array}{c} R_{p}\left(“obj”\right)=-lnP_{r}\left(I_{p}|O\right),\\ R_{p}\left(“\text{bkg}”\right)=-lnP_{r}\left(I_{p}|B\right), \end{array}\right) \end{array}$$

(3) $$\begin{array}{c} \delta \left(\right)l_{p},l_{q}\left(\right)=\left\{\begin{array}{cc} 1, & l_{p}\neq l_{q},\\ 0, & l_{p}=l_{q}. \end{array}\right) \end{array}$$

In equations (2) and (3), *λ* expressed the weighted factor; *N* stood for the collection of pixel points; *p* and *q* represented any pixel points in *N*; *I* meant the gray value; and *A* stood for the discontinuous penalty.

In order to solve the deficiencies of traditional Graph Cuts algorithm that required manual setting of foreground and background markers, automatic generation of threshold markers was for improvement in this study, so as to be more suitable for bone tissue CT image segmentation. Firstly, there was format conversion, and the DICOM file of medical image was converted into bitmap for the convenience of subsequent processing. Then, the regional and boundary items were established. The weight of *n*-links edge was very critical for the image segmentation quality, so it was necessary to consider not only the pixel position relationship between the two endpoints, but also the pixel difference value. The weight calculation method based on gray scale and distance was expressed as follows:

(4) $$\begin{array}{c} A_{\left\{p,q\right\}}=\exp\left(-\frac{{\left(I_{p}-I_{q}\right)}^{2}}{2\sigma^{2}}\right)\cdot \frac{1}{\text{dist}\left(p,q\right)}, \end{array}$$

where dist(*p*, *q*) stood for distance from the pixel *q* to the pixel *p*.

The model shown in equation (2) was still used for the setting of regional item. After threshold segmentation was processed, there were three types of images (Label-BackGround, Label-Object, and pixel points to be segmented). The network diagram was established, and the regional and boundary items corresponded to t-links and *n*-links, respectively. The maximum flow/minimum segmentation algorithm was adopted to seek the solution, so as to obtain the initial segmentation results. At this time, most foreground and background points could be identified, and the marking errors caused by small differences between foreground and background in some regions could be corrected manually.

In order to deal with threshold selection difficulty and noise sensitivity in the above algorithm, the morphological marker automatic generation method was adopted to optimize the algorithm. Open operation and closed operation were two crucial operations in morphology. Open operation could reduce image noise to make contour boundary smoother. The horizontal direction was of 1 *∗* 3 structural elements, morphological opening was applied to get the initial mark image, and the mark point image with the original image was input to the Graph Cut algorithm. The maximum flow/minimum segmentation algorithm was adopted to improve the initial segmentation, there was judgment for initial segmentation image quality, and there was manual modification by combining with man-machine interaction for continuous iteration until there was no segmentation error. The specific process is shown in Figure 1.

### 2.5. Evaluation of Therapeutic Effects

VAS was employed to assess the pain degree of knee joint. The pain degrees of patients were graded by themselves based on their own pain conditions, and the score ranged from 0 to 10. In addition, the pain degree increased gradually from 0 to 10 (0 meant no pain and 10 stood for the most severe pain).

The Roles and Maudsley (RM) scale was applied to assess the physical activity of patient. It included 4 grades, namely, excellent, good, general, and poor, corresponding to 1, 2, 3, and 4 points, respectively. There was 1 point if the patient had no pain during exercise and in normal life. The patient sometimes felt pain during exercise and in normal life, so there were 2 points. If the patient felt pain after a little activity, it was 3 points. If the patient was unable to do normal activities, the score was 4 points.

The Western Ontario and McMaster Universities osteoarthritis index (WOMAC) and Lequesne index scales were adopted to assess the body function of patient. The WOMAC score scale included pain, joint function, and stiffness. There were 5 ratings including difficult, mild, medium, very, and extreme that corresponded to 0, 1, 2, 3, 4, and 5 points in sequence. The Lequesne index scale involved tenderness, swelling, morning stiffness, walking ability, knee joint exercise pain, and rest pain, with 0, 1, 2, and 3 points for each aspect.

### 2.6. Quality Nursing Intervention

All patients were treated with high-quality nursing intervention after surgery, and the nursing effect was evaluated by SSS. First, the head nurse was selected as the group leader to set up a nursing team and reasonably arrange the nursing work and specific division of labor of the staff within the group, so as to ensure that the nursing staff were on duty 24 hours a day and give comprehensive and meticulous care to each patient.

The drug therapy included was as follows: 2 mL of sodium hyaluronate was injected into the articular cavity of the patient 1–2 times a week for a total of 6 weeks. If the patient suffered from severe pain, external application could be made with dressings of activating blood circulation and dissipating blood stasis. If the patient was well tolerated and in good condition, the traditional Chinese medicine with activating blood circulation to dissipate blood stasis could be adopted as adjuvant therapy.

The rehabilitation exercise was as follows. According to the condition of patient, the nursing staff should guide and help the patient to do some rehabilitation exercises, such as limb stretching and limb twisting. In addition, there was also appropriate massage, foot bath, and physical therapy to improve the symptoms of pain and swelling and promote the recovery of patients.

### 2.7. Statistical Analysis

SPSS20.0 statistical software was used for analysis, the measurement data were expressed as mean ± standard deviation ($\bar{x}\pm s$), and there was the pairwise comparison analyzed by one-way variance (ANOVA) and tested by least significant difference (LSD). Besides, *χ*^2^ test was used for pairwise comparison and analysis of count data. If *P* < 0.05, there was a statistically substantial difference.

## 3. Results

### 3.1. Computed Tomography Imaging Segmentation Results Based on Image Segmentation Algorithm

Dice similarity coefficient was employed to evaluate the segmentation results of different algorithms, and the definition of Dice similarity coefficient was expressed as follows:

(5) $$\begin{array}{c} \text{Dice}\left(M,N\right)=\frac{2\left|M\cap N\right|}{\left|M\right|+\left|N\right|}. \end{array}$$

In equation (5), *M* and *N* stood for the image pixel set obtained by the gold standard and the segmentation algorithm, respectively.

Figures 2 and 3 indicated the segmentation results of different algorithms. The Dice similarity coefficients of the traditional Graph Cuts algorithm, threshold + Graph Cuts algorithm, and morphology + Graph Cuts algorithm were 0.528, 0.854, and 0.926, respectively, and the running time was 0.112 seconds, 0.045 seconds, and 0.069 seconds in sequence. Dice similarity coefficient ranged within 0-1, and the larger the value was, the smaller the gap between algorithm segmentation and standard segmentation was. According to the above results, the segmentation quality and algorithm efficiency of morphology + Graph Cuts algorithm were more excellent.

CT images of patients with KOA were segmented by different segmentation algorithms, as shown in Figure 4. The number of seed points required by the traditional Graph Cuts algorithm was large but its segmentation effect was poor. Threshold + Graph Cuts algorithm segmentation was more accurate, but there were holes and isolated points. Compared with the traditional Graph Cuts algorithm and threshold + Graph Cuts algorithm, the morphology + Graph Cuts algorithm had the best segmentation effect on CT images.

### 3.2. Clinical Data of Patients with KOA from Both Groups

Table 1 showed the comparison results of clinical data of patients with KOA from groups A and B. In group A, there were 22 male and 20 female patients with KOA, with an average age of 53.14 ± 10.39 years, an average height of 165.23 ± 8.98 cm, an average weight of 67.87 ± 4.36 kg, and the body mass index (BMI) of 24.36 ± 1.54 kg/m^2^. Furthermore, there were 20 male and 18 female patients with KOA in group B, with an average age of 54.03 ± 9.76 years, an average height of 167.24 ± 8.02 cm, an average weight of 68.36 ± 5.02 kg, and the BMI of 23.98 ± 1.25 kg/m^2^. There were no statistically obvious differences in gender, age, height, weight, and BMI of patients with KOA from groups A and B (*P* > 0.05).

### 3.3. Comparison of Knee Joint Pain Improvement among Patients in the Two Groups

Figure 5 revealed the comparison of VAS scores of KOA patients from both groups before and after treatment. VAS scores of patients in group A were 5.95 ± 1.09 points, 4.78 ± 0.52 points, 2.76 ± 0.55 points, and 1.92 ± 0.67 points before treatment, after treatment, 1 month after treatment, and 3 months after treatment, respectively. Moreover, VAS scores of patients from group B were 6.09 ± 1.15 points, 5.15 ± 0.80 points, 2.72 ± 0.78 points, and 1.56 ± 0.54 points before treatment, after treatment, 1 month after treatment, and 3 months after treatment in turn. VAS scores after treatment of patients in both groups A and B decreased in contrast to those before treatment, and the difference was statistically substantial (*P* < 0.05). VAS scores after treatment and 3 months after treatment of patients in group B reduced sharply in contrast to the scores of group A (*P* < 0.05).

### 3.4. Comparison on Knee Joint Function Improvement of Patients with KOA from the Two Groups

There were the comparison results of RM scores of patients in groups A and B before and after treatment (Figure 6). The RM scores of patients in group A were 3.26 ± 0.77 points, 2.45 ± 0.59 points, 1.71 ± 0.62 points, and 1.24 ± 0.47 points before treatment, after treatment, 1 month after treatment, and 3 months after treatment in sequence. In addition, RM scores of patients in group B before treatment, after treatment, 1 month after treatment, and 3 months after treatment were 3.25 ± 0.72 points, 3.25 ± 0.72 points, 1.42 ± 0.48 points, and 1.11 ± 0.32 points, respectively. RM scores of patients in groups A and B decreased after treatment compared with those before treatment, and there was a statistically remarkable difference (*P* < 0.05). RM scores of KOA patients from group B were steeply lower than the scores of group A after treatment and 1 month after treatment (*P* < 0.05).

The WOMAC scores of patients with KOA in groups A and B were compared before and after treatment as shown in Figure 7. WOMAC scores of patients in group A before treatment, after treatment, 1 month after treatment, and 3 months after treatment were 56.94 ± 10.87 points, 49.20 ± 10.23 points, 38.87 ± 8.35 points, and 32.54 ± 7.12 points, respectively. Besides, WOMAC scores of patients in group B were 57.45 ± 10.23 points, 49.02 ± 11.25 points, 31.64 ± 9.15 points, and 24.27 ± 7.27 points, respectively, before treatment, after treatment, 1 month after treatment, and 3 months after treatment. WOMAC scores of all patients from groups A and B after treatment reduced dramatically in contrast to those before treatment (*P* < 0.05). In addition, WOMAC scores of patients with KOA from group B were sharply lower than scores of group A 1 month and 3 months after treatment (*P* < 0.05).

Figure 8 expresses the comparison results of Lequesne index scores of patients from groups A and B before and after treatment. The Lequesne scores of patients in group A before treatment, after treatment, 1 month after treatment, and 3 months after treatment were 15.06 ± 4.52 points, 14.55 ± 3.85 points, 10.77 ± 3.91 points, and 8.46 ± 2.17 points in turn. What is more, Lequesne scores of patients in group B before treatment, after treatment, 1 month after treatment, and 3 months after treatment were 15.08 ± 4.22 points, 13.74 ± 3.13 points, 9.56 ± 3.42 points, and 6.05 ± 2.07 points, respectively. Lequesne scores of patients in groups A and B dropped after treatment by comparing with those before treatment, and the difference was statistically marked (*P* < 0.05). The Lequesne score of patients in group B 3 months after treatment was markedly lower than the score of group A (*P* < 0.05).

### 3.5. Comparison on Adverse Reactions of KOA Patients in Groups A and B

During the treatment, 3 cases of group A and 1 case of group B showed mild redness and swelling, which disappeared after local cold application for 24 hours. Furthermore, 1 patient in group B was unbearable for the pain, so the treatment was stopped immediately, and the pain was gradually eased after the patient rested for 1 hour. The comparison results of the adverse reaction rate of KOA patients in the two groups are shown in Figure 9. Besides, the adverse reaction rates of patients in groups A and B were 7.1% and 4.8% in turn. There were no statistically great differences in the adverse reaction rates of KOA patients from the two groups (*P* > 0.05).

### 3.6. Comparison on Nerve Function Rehabilitation of KOA Patients in the Two Groups

The comparison results of SSS scores of patients in groups A and B before and after nursing are shown in Figure 10. In group A, SSS score of patients before nursing was 34.69 ± 3.13 points and that after nursing was 28.15 ± 1.98 points. Before and after nursing, SSS scores of patients with KOA from group B were 34.72 ± 3.09 points and 16.35 ± 2.12 points, respectively. Thus, SSS scores of patients in groups A and B were compared before nursing, suggesting that the difference was not statistically remarkable (*P* > 0.05), while the SSS scores of patients from group B after nursing were dramatically lower than the scores of group A (*P* < 0.05).

## 4. Discussion

ISA was applied to improve and optimize the segmentation effect of medical images, and the results showed that the morphology + Graph Cuts algorithm had the best segmentation effect on CT images in contrast to the threshold + Graph Cuts algorithm and traditional Graph Cuts algorithm. This was consistent with the research results of Wu et al. [13], indicating that the CT segmentation method based on ISA could promote the segmentation accuracy of medical CT images. KOA is the leading cause of chronic bone and muscle pain. In recent years, RSWT has been employed to treat patients with KOA. In this study, there was a comparison on the curative effect of ultrasound treatment and RSWT for KOA. It was found that VAS scores before and after treatment were extremely different among KOA patients in the two groups, and the pain degree of patients in group B decreased hugely by comparing with the degree of group A (*P* < 0.05). This suggested that both ultrasound therapy and RSWT could help patients with pain symptoms, and RSWT was more effective. This was in accordance with the research results of Lee et al. [14] and Kang et al. [15]. The knee joint function rehabilitation of KOA patients was evaluated by RM, WOMAC, and Lequesne index scores in this study, and it was found that there were statistically marked differences in the RM, WOMAC, and Lequesne index scores of patients in groups A and B before and after treatment (*P* < 0.05). With the extension of treatment time, RM, WOMAC, and Lequesne index scores decreased gradually (*P* < 0.05). Therefore, the knee joint function of patients in group B was obviously better than that of group A (*P* < 0.05). There was no statistically great difference in the adverse reaction rates of patients in the two groups (*P* > 0.05). Lizis et al. [16] pointed out that the WOMAC and ROM scores of KOA patients treated with RSWT were superior to those of KOA patients treated with kinesitherapy (KIN) by comparing the influences of RSWT and KIN for KOA patients. The research findings of Zhong et al. [17] reflected that VAS, WOMAC, and Lequesne index scores of KOA patients with RSWT were extremely better than those of KOA patients with placebo at the 5th and 12th week (*P* < 0.05). Moreover, all the patients showed improvement in pain and disability scores during 12 weeks of follow-up (*P* < 0.05), the adverse reaction rates of them were similar, and there were no serious side effects. This was consistent with the research results of this study. In this study, high-quality nursing was used for intervention treatment, and it was found that the SSS scores of nerve function rehabilitation after nursing in patients of group B were steeply lower than the scores of group A (*P* < 0.05). To some extent, it revealed that RSWT could promote tissue repair, thus contributing to nerve function rehabilitation. Based on the above results, RSWT had a better effect on alleviating pain and improving knee joint function in KOA patients.

## 5. Conclusion

The ISA-based CT imaging technology was for analysis of curative effects on KOA. It was found that RSWT had a more marked clinical effect, which could effectively relieve patients' pain and promote the knee joint and nerve function rehabilitation, and it was better than that of ultrasonic treatment through the analysis of the pain symptoms and knee joint and nerve function rehabilitation in patients with KOA before and after treatment. However, there were still some deficiencies in this study; for example, the sample size was limited, there was evaluation of only 3 months, and there was a lack of long-term efficacy evaluation. In the future, the number of samples and observation time should be increased to assess the long-term efficacy, so as to further analyze the therapeutic effects of KOA. In summary, the results of this study could provide reference for the imaging diagnosis and treatment of KOA.

## Figures and Tables

**Figure 1:** Flowchart of morphological marker graph cut algorithm.

**Figure 2:** Comparison of Dice similarity coefficient among different algorithms.

**Figure 3:** Comparison of running time among different algorithms.

**Figure 4:** CT image segmentation results of different segmentation algorithms: (a) The source image, (b) The image of Graph Cuts algorithm, (c) The image of threshold + Graph Cuts algorithm, and (d) The image of morphology + Graph Cuts algorithm.

**Figure 5:** Comparison on VAS scores of patients with KOA from both groups before and after treatment. *Note*. ^*∗*^ indicated *P* < 0.05 compared with before treatment; and ^#^ meant *P* < 0.05 in contrast to group A.

**Figure 6:** Comparison on RM scores of KOA patients from groups A and B before and after treatment. *Note*. ^*∗*^ indicated *P* < 0.05 compared to before treatment; and ^#^ showed *P* < 0.05 in contrast to group A.

**Figure 7:** Comparison on WOMAC scores of KOA patients from groups A and B before and after treatment. *Note*. ^*∗*^ showed that there was a statistically obvious difference compared to before treatment (*P* < 0.05); and ^#^ indicated that there were statistically considerable differences in contrast to group A (*P* < 0.05).

**Figure 8:** Comparison on Lequesne scores of KOA patients from groups A and B before and after treatment. *Note*. ^*∗*^ showed that there was a statistically substantial difference compared with before treatment (*P* < 0.05); and ^#^ indicated that there were statistically marked differences in contrast to group A (*P* < 0.05).

**Figure 9:** Comparison on adverse reaction rates of KOA patients in groups A and B.

**Figure 10:** Comparison on SSS scores of KOA patients in the two groups. *Note*. ^#^ indicated that the difference was statistically obvious in contrast to group A (*P* < 0.05).

**Table 1:** Comparison on clinical data of all patients in both groups.

	Group A (*n* = 42)	Group B (*n* = 42)	*P*
Gender (male/female)	22/20	24/18	0.123
Age (years old)	53.14 ± 10.39	54.03 ± 9.76	0.113
Height (cm)	165.23 ± 8.98	167.24 ± 8.02	0.097
Weight (kg)	67.87 ± 4.36	68.36 ± 5.02	0.068
BMI (kg/m^2^)	24.36 ± 1.54	23.98 ± 1.25	0.612

## Data Availability

The data used to support the findings of this study are available from the corresponding author upon request.
